The article "Multiresolution-Based Singular Value Decomposition Approach for Breast Cancer Image Classification" was retracted in 2024. Reasons: signs of a paper mill; suspected computer-generated content; unreliable results or conclusions; concerns about the data.

# Multiresolution-Based Singular Value Decomposition Approach for Breast Cancer Image Classification

**DOI:** 10.1155/2022/6392206

**Published:** 2022-08-11

**Authors:** Suman Mann, Amit Kumar Bindal, Archana Balyan, Vijay Shukla, Zatin Gupta, Vivek Tomar, Shahajan Miah

**Affiliations:** ^1^Department of Information Technology, Maharaja Surajmal Institute of Technology, New Delhi, India; ^2^Department of Computer Science & Engineering, MM Engineering College, MMDU, Mullana, Ambala, India; ^3^Department of Electronics and Communication Engineering, Maharaja Surajmal Institute of Technology, New Delhi, India; ^4^Department of Computer Science & Engineering, Greater Noida Institute of Technology, Greater Noida, India; ^5^School of Computing Science & Engineering, Galgotias University, Greater Noida, Gautam Buddh Nagar, Uttar Pradesh, India; ^6^Department of Computer Science & Engineering, KIET Group of Institutions, Delhi-NCR, Ghaziabad, Uttar Pradesh, India; ^7^Department of EEE, Bangladesh University of Business and Technology (BUBT), Dhaka, Bangladesh

## Abstract

Breast cancer is the most prevalent form of cancer that can strike at any age; the higher the age, the greater the risk. The presence of malignant tissue has become more frequent in women. Although medical therapy has improved breast cancer diagnostic and treatment methods, still the death rate remains high due to failure of diagnosing breast cancer in its early stages. A classification approach for mammography images based on nonsubsampled contourlet transform (NSCT) is proposed in order to investigate it. The proposed method uses multiresolution NSCT decomposition to the region of interest (ROI) of mammography images and then uses Z-moments for extracting features from the NSCT-decomposed images. The matrix is formed by the components that are extracted from the region of interest and are then subjected to singular value decomposition (SVD) in order to remove the essential features that can generalize globally. The method employs a support vector machine (SVM) classification algorithm to categorize mammography pictures into normal, benign, and malignant and to identify and classify the breast lesions. The accuracy of the proposed model is 96.76 percent, and the training time is greatly decreased, as evident from the experiments performed. The paper also focuses on conducting the feature extraction experiments using morphological spectroscopy. The experiment combines 16 different algorithms with 4 classification methods for achieving exceptional accuracy and time efficiency outcomes as compared to other existing state-of-the-art approaches.

## 1. Introduction

Breast cancer is now one of the most common cancers in women. According to the World Health Organization, between 2008 and 2012, breast cancer incidence and mortality have increased by approximately 20% and 14% [1]. Faced with the increasingly severe health situation, technical workers from self-detection activity to medical image-based breast cancer early detection techniques, especially the study of mammograms, manage breast cancer mortality to some extent. However, by X-ray, some of the mammary images obtained by photography will inevitably contain some noise, such as fatty breast groups that are very close to the gray level of the lesion area organization; it is difficult even for experienced radiologists to accurately identify the type of tumor (benign, malignant, and normal) [2, 3], and in dense breast cases, patients with this type of breast are usually young patients. It can be seen that the research on the classification of adipose breast cancer tumors has strong practical application value and social value.

The article "Multiresolution-Based Singular Value Decomposition Approach for Breast Cancer Image Classification" was retracted in 2024. Reasons: signs of a paper mill; suspected computer-generated content; unreliable results or conclusions; concerns about the data.

At present, the classification methods based on mammography images are demonstrated as follows: (1) Feng et al. proposed a method for detecting lesions based on region growth [4]; (2) Hmaidan et al. used Z-moments as the shape which is one of the methods of a shape descriptor [5]; (3) Orel et al. adopted the salient index number to represent the geometry of the lesion boundary [6]; (4) Burriel et al. adopted the strategy of convolutional neural network (CNN) segmentation in the feature extraction stage [7]; and (5) detection and classification by wavelet transform were proposed by researchers and highlight the different methods of mammography.

Because mammograms do not show perfectly the swelling of the outline of the tumor, the first four mentioned above are the most important for classifying the tumor. Both methods require the doctor to manually assign the tumor region to each image. The fifth method proposed by Sidney et al. does not require a manual, but the original breast image is decomposed into a series of subimages with different spatial resolutions and frequency characteristics, reflecting the local variation features of the original breast images. Thus, various feature information can be extracted from different subimages using Z-moments, but the wavelet transform has only three directions of horizontal, vertical, and diagonal detail information and subsamples the original breast image. Therefore, it has a great impact on the contours and linear features of the original breast image. The singularity of the surface is difficult to express well [8].

As an important factor affecting the experimental effect, the classification method choosen should be a good classification method for breast images. Correct classification is the key to the success of the experiment. The obtained experimental data were tested with different classification methods, and the results are compared. It is found that the linear kernel function of support vector machines (SVM) has the best classification effect. But authors did not perform any cleaning work on their data; as a result, the amount of data is large and complex, so choosing a good data cleaning method is also very important.

The article "Multiresolution-Based Singular Value Decomposition Approach for Breast Cancer Image Classification" was retracted in 2024. Reasons: signs of a paper mill; suspected computer-generated content; unreliable results or conclusions; concerns about the data.

Because of the mentioned issues, this paper proposes the nonsubsampled contourlet transform (NSCT) method for classifying mammography images. Pretreated lipid NSCT image decomposition of the fatty mammogram is performed to obtain the original breast image. A series of sub images are extracted from the gland image through Z-moments in order to extract features from a large amount of data using the method of value decomposition (singular value decomposition (SVD)) is performed. After cleaning, different classification methods are used to classify them, so it not only reduces the amount of data but also improves the quality of data, making the classification more accurate. Both the accuracy and time efficiency are better than those of the method proposed by previous researchers.

The organization of this paper is as follows: Section 2 is the premap of mammography images which is the preprocessing process; Section 3 introduces the framework of this method; Section 4 is divided into three parts: the first part introduces the nonsubsampling contour transformation method (NSCT) principle and its applications, the second part presents Z-moments, and the third part discusses the classification algorithm of SVM; Section 5 introduces the experimental dataset and presents the experimental results and analysis; and Section 6 presents the conclusion and scope for future work.

## 2. Preprocessing Process

The following main studies apply mathematical morphology to the mammography image method for preprocessing.

Mathematical morphology is a nonlinear filtering method in image processing. It has four basic operations: dilation, erosion (or invasion eclipse), opening, and closing, which are different in binary and grayscale image features [9–12]. Based on these methods, many mathematical forms can be combined and algorithms can be used to analyze the shape and structure of images for analytical processing, including image segmentation, feature extraction, boundary detection, image filtering, and image enhancement and restoration.

Equations (1) and (2) are corrosion and dilation, respectively, in mathematical expression:

(1) $$\begin{array}{c} \xi_{g}\left(f\right)\left(u\right)=\underset{v\in S}{⋂}f\left(v\right)⋁\bar{g}\left(u-v\right), \end{array}$$

(2) $$\begin{array}{c} \xi_{g}\left(f\right)\left(u\right)=\underset{v\in S}{⋃}f\left(v\right)⋁g\left(u-v\right), \end{array}$$

where *f* : *S*⟶[0, 1] and *g* : *S*⟶[0, 1] are normalized single spectral images, *S*⊆*Z*^2^, the symbols ⋃ and ∨ are associated with the max operation, the symbols ⋂ and ∧ are associated with the min operation, and $\bar{g}\left(u\right)=1-g\left(u\right)$. For ∀*u* ∈ *S*, *g* : *S*⟶[0, 1] are the corresponding erosion and dilation structuring elements [9–12].

The article "Multiresolution-Based Singular Value Decomposition Approach for Breast Cancer Image Classification" was retracted in 2024. Reasons: signs of a paper mill; suspected computer-generated content; unreliable results or conclusions; concerns about the data.

Combining the mathematical expressions for erosion and dilation, one can get open. The mathematical expression *γ*_*g*_(*f*)(*u*) uses the original erosion-and-dilation reason. Next, consider the normalized single spectral image *f* : *S*⟶[0, 1] by the structure element *g* : *S*⟶[0, 1], the remaining area generated by the *k*th opening operation. The mathematical expression for (*k* ≥ 0) is

(3) $$\begin{array}{c} V\left(k\right)=\underset{v\in S}{\sum }\gamma_{g}^{k}\left(f\right)\left(u\right). \end{array}$$

Through the above description of the basic operations of mathematical morphology, expression (4) is obtained (the discrete cumulative density function):

(4) $$\begin{array}{c} E\left[k\right]=1-\frac{V\left(k\right)}{V\left(0\right)}. \end{array}$$

The discrete density function, also known as mode spectrum or morphological spectrum, is described by equation (5) [12]. Learning about its preservation through morphological theory proves that each binary image has a unique representation based on that spectrum because this pattern or morphological spectrum can be used as an exact shape-based feature extractor and the mode spectrum has negligible mammary irregularities at the edges of the mass leading to low-amplitude changes in the morphological spectrum ability and its ability to function as a tumor regardless of tumor size which is nothing but a unique representation of a shape. This is the reason for the preprocessing method of the adrenal X-ray images. Reflecting the histopathological complexity of adrenal glands, the classification of adrenal lesions may be complex [13–15]. Lesions of the adrenal gland can be roughly classified as either primary or secondary. Primary adrenal lesions, that is, lesions originating from the adrenal gland itself, can be cortical or medullary in origin. Lesions of the adrenal glands can also be classified according to their laterality, that is, as unilateral or bilateral [16]. Additionally, bilateral lesions might develop with syndromes of hormone excess or insufficiency. It complements functional imaging and hormonal analysis in the diagnosis of functioning tumors [17]. The role of adrenal X-ray imaging is to differentiate between benign and malignant lesions and to provide diagnosis wherever possible [18].

(5) $$\begin{array}{c} \xi_{g}\left[k\right]=E\left[k+1\right]-E\left[k\right]. \end{array}$$

To calculate the morphological spectrum of an image, one has to perform equation (5) until the algorithm converges. Different mammograms in the database at different times of iterative calculations are required to obtain the morphological spectral results in order to avoid the problem of different morphological spectrum sizes; 7 systems will be used as metrics to represent these spectra, i.e., mean, standard deviation, mode, median value, kurtosis, min, and max.

The article "Multiresolution-Based Singular Value Decomposition Approach for Breast Cancer Image Classification" was retracted in 2024. Reasons: signs of a paper mill; suspected computer-generated content; unreliable results or conclusions; concerns about the data.

## 3. Introduction to the Framework

The following describes the feature extraction and classification framework.

Methods for classifying breast lesions from mammography images are highly dependent on the feature extraction stage. This paper uses a hybrid approach that combines NSCT and Z-moments. The overall framework of the feature extraction method is shown in Figure 1. The combination of multiresolution NSCT and Z-moments can be mixed. Texture and shape features are used to improve image representation in the classification stage.

Mammography is the preferred method for early detection of breast cancer; nevertheless, only a few specialists have difficulties interpreting mammography images [19]. Classification of mammography images to normal, benign, and malignant is highly dependent on the feature extraction stage which is done through the NSCT method [20]. Feature extraction is done in two stages: in the first stage, the region of interest as an input image for subsampled pyramid filter banks (NSPFB) is decomposed into low-pass subband images (LSI) and bandpass subband image (BSI) to achieve multiscale decomposition of the image [21]. Then, the nonsubsampled directional filter bank (NSDFB) is used to decompose the BSI into the multidirectional subband image and use the bandpass directional subband image (BDSI), so that the multidirectional decomposition of the image can be realized for mathematical morphology, and the procedure is repeated.

The operation is to obtain a multilayer NSCT of the input image [22] which is a raw breast. The X-ray image is decomposed by the NSPFB to the first scale in order to get the images LSI1 and BSI2. Then, the image is obtained by NSPFB decomposition of the second scale LSI2 and BSI2 and so on.

If BSI*n* (*n* ∈ 1, 2, ⋯, *n*) is decomposed in the *m*-level direction; that is, 2 m *m*-level BDSIs with the same size as the original image can be obtained, called for BDSIm. The original X-ray image can be decomposed by *J*-slice NSCT. Get 1 LSI*J* and ∑_*j*=1_^*J*^2^*m*_*j*_^ BDSIs, where *m*_*j*_ is the scale *j* direction series below.

The article "Multiresolution-Based Singular Value Decomposition Approach for Breast Cancer Image Classification" was retracted in 2024. Reasons: signs of a paper mill; suspected computer-generated content; unreliable results or conclusions; concerns about the data.

According to the above description, several concepts can be defined here:

**Definition 1 (low-pass subband image (LSI)).**

(6) $$\begin{array}{c} \text{LSI}i=H0\left(\text{LSI}\left(i-1\right)\right),\;i\in \left\{1,2,\cdots \right\}, \end{array}$$

where LSIi represents the LSI decomposed by the *i*th scale NSPFB, and when *i* = 1, LSI0 represents the original mammogram; the function *H*0(*z*) is the bandpass decomposition of the two-channel nonsubsampling filter bank (NSPFB) waver.

**Definition 2 (bandpass subband image (BSI)).**

(7) $$\begin{array}{c} \text{BSI}i=H1\left(\text{LSI}\left(i-1\right)\right),\;i\in \left\{1,2,\cdots \right\}, \end{array}$$

where BSIi represents the BSI decomposed by the *i*th scale NSPFB, and when *i* = 1, LSI0 represents the original mammogram; the function *H*1(*z*) is the bandpass decomposition of the two-channel nonsubsampled filter bank (NSPFB) waver.

According to the above description and previous research results, this multipoint high-resolution image decomposition method can effectively detect breast lesions, suspicious lesions, and breast tissue successfully [22].

The second stage will use the Z-moments obtained in the first stage; the subgraph of the feature extraction method has been widely used in the shape analysis of lesions [6, 23] because the shape is important for determining breast cancer lesions; the degree of malignancy is critical [24]. For every raw milk, 32 high-dimensional subimages are extracted from the decomposition of the gland X-ray image, so a raw mammogram can be extracted to 480 eigenvalues, as shown in Figure 1.

Finally, the extracted 480 eigenvalues are decomposed by SVD for feature reduction to obtain features with smaller dimensions but can generalize the global quality. Because the learning of a classifier is typically a time-consuming process that may entail numerous iterations of training data [25], cross-validation paired with different random beginning conditions and testing of various kernels (learning functions) were carried out, and the more significant the amount of data, the more time-consuming it will be. Therefore, the SVD method is used in this paper to extract essential features that can generalize globally, thereby reducing the amount of data and time consumption.

The above is an introduction to the framework shown in Figure 1, and compared with the state-of-the-art methods, it achieves both accuracy and time efficiency with remarkable result.

## 4. Feature Extraction Stage

The process of feature extraction is based on NSCT and the construction of Z-moments and the classification algorithm flow of SVM.

The article "Multiresolution-Based Singular Value Decomposition Approach for Breast Cancer Image Classification" was retracted in 2024. Reasons: signs of a paper mill; suspected computer-generated content; unreliable results or conclusions; concerns about the data.

### 4.1. Feature Extraction Based on NSCT

NSCT was proposed by Cunha et al. in 2005. Shift-invariant contour transform [26] is based on NSPFB, and NSDFB transformation of both methods is described in detail below.

### 4.2. Nonsubsampling Tower Filters

The nonsubsampling tower filter (NSPFB) differs from a number proposed by Do and Veterli that can better represent two-dimensional signals (learning tools—Laplacian pyramid (LP) multiscale analysis in the contour transformation method) [27]. Because of LP multiscale segmentation, both analysis and discrete wavelet transform are used when decomposing the original mammogram. Using downsampling, results in multiscale decomposition of low-frequency images and high-frequency images do not have the size of the original image. The downsampling process will be distorted in the filter, so using LP multiscale, neither the solution nor the discrete wavelet transforms lack translation invariance. While the NSPFB cancels the downsampling operation of the signal during its decomposition, the wave filter performs the corresponding upsampling (interpolation) operation, reducing the original milk distortion of glandular radiographs during multiscale decomposition.

Figure 2 shows the decomposition process of a three-layer NSPFB [27]. As can be seen from Figure 2, each mammogram is processed by NSPFB. Decompose it into images of different scales. The first scale decomposition gets LSI1 and BSI1, the second scale decomposition gets LSI2 and BSI2, and so on.

#### 4.2.1. Nonsubsampling Directional Filters

The nonsubsampling directional filter (NSDFB) is a two-channel filter bank, whose main function is to perform the BSI obtained by NSPFB tree structure decomposition. And if the BSI passes through an *l*-ary tree structure decomposition, effectively divide the signal into 2*l* subbands whose frequency bands are divided into wedges. The discrete wavelet transform can also perform this process, but it is far from scatter wavelet transform which can only extract detail images in horizontal, vertical, and diagonal directions, while NSDFB can extract detail images in multiple directions. Each orientation sub map obtained by NSDFB is larger than the original breast image and is same as all bandpass divisors which is different from the discrete wavelet transform. The sum of the images is equal to the original image.

**Definition 3 (band pass direction subband image (BDSI)).**

(8) $$\begin{array}{c} \text{BDSI}1=\left\{U_{0}\left(\text{BSI}j\right)+U_{1}\left(\text{BSI}j\right)\right\},\;\;j=\left\{1,2,\cdots \right\}. \end{array}$$

This means that a 1-level directional decomposition of BSI*j* will result in 2 BDSI1s.

The article "Multiresolution-Based Singular Value Decomposition Approach for Breast Cancer Image Classification" was retracted in 2024. Reasons: signs of a paper mill; suspected computer-generated content; unreliable results or conclusions; concerns about the data.

BSI*j* represents the BSI decomposed by the *j*th scale NSPFB. BSI*j* performs 2-level directional decomposition; then, 4 BDSI2 are obtained, whose expression formula is

(9) $$\begin{array}{c} \text{BDSI}2=\left\{\begin{array}{c} \left.U_{0}\left(U_{0}\left(\text{BSI}j\right)\right)\right)+U_{1}\left(U_{0}\left(\text{BSI}j\right)\right)+\\ \left.U_{0}\left(U_{1}\left(\text{BSI}j\right)\right)\right)+U_{1}\left(U_{1}\left(\text{BSI}j\right)\right) \end{array}\right\},\;j\in \left\{1,2,\cdots \right\}. \end{array}$$

The decomposition of BSI*j* in the *m*-level direction is carried out and so on.

As shown in Figure 3, it is shown that different methods are used for different scales of BSI, the process of decomposition; because BSI1 is compared with other BSI*i* (*i* ≠ 1), in its graph, the structure, outline, and texture of the image are the clearest, and the details of the original image are more clear. It is similar, so it is decomposed in 3-level direction to get 8 BDSI3; BSI2 performs 2-level tree structure decomposition to obtain 4 BDSI2 and BSI3.

Perform 1-level tree structure decomposition to get 2 BDSI1, and the last LSI3, which is most similar to the original image, does not perform tree-like segmentation solution; the Zernike moment can be directly constructed [27].

### 4.3. Constructing Zernike Moments

LSI3 and all BDSI1 and both BDSI2 and BDSI3 are used to construct Z-moments. Enter an image. Each original image expanded after being decomposed by NSCT has 15 subgraphs, and each subgraph can be constructed with 32 Z-moments of the value. The calculation process of Z-moments consists of 3 steps: calculation of radial polynomial, calculation of Zernike basis functions, and calculation of Z-moments that project images onto Zernike basis functions.

The process of obtaining Z-moments starts at Zernike calculation of radial polynomials. Real-valued one-dimensional radial polynomial *R*_*n*,*m*_ is defined as

(10) $$\begin{array}{c} R_{n,m}=\overset{\left(n-\left|m\right|\right)/2}{\underset{s=0}{\sum }}{\left(-1\right)}^{s}\frac{\left(n-s\right)!}{s!\left(\left(n-\left|m\right|\right)/2-s\right)!\left(\left(n-\left|m\right|\right)/2-s\right)!}\rho^{n-2s}, \end{array}$$

where *n* is a nonnegative integer; *m* is an integer such that *n* − ∣*m* | = even number and |*m* | ≤*n*; and *ρ* is the length from the origin to the vector (*x*, *y*).

According to formula (10), the complex-valued two-dimensional Zernike defined by the unit circle basis function is

(11) $$\begin{array}{c} V_{n,m}\left(\rho ,\theta \right)=R_{n,m}\left(\rho \right)e^{jm\theta },\;\left|\rho \right|\leq 1. \end{array}$$

The complex-valued two-dimensional Zernike polynomials satisfy the following orthogonal conditions:

(12) $$\begin{array}{c} \int_{0}^{2\pi }\int_{0}^{1}V_{n.m}^{*}\left(\rho ,\theta \right)V_{p,q}\left(\rho ,\theta \right)\rho d\rho d\theta =\left\{\begin{array}{cc} \frac{\pi }{n+1},n=p, & m=q,\\ 0, & \text{else}. \end{array}\right. \end{array}$$

Among them, ∗ represents a conjugated complex number. As mentioned earlier, orthogonality means that the image information of different moments formed by different *n* and *m* combinations is nonredundant. The rest are nonoverlapping. Using this property, the contribution from every combination is made unique and invariant of the data in the image [28]. In fact, different combinations exist. All features have the same importance. In a composite of *n*, *m* Z-moments are defined as

(13) $$\begin{array}{c} Z_{n,m}=\frac{n+1}{\pi }\int_{0}^{2\pi }\int_{0}^{1}f\left(\rho ,\theta \right)V_{n,m}^{*}\left(\rho ,\theta \right)\rho d\rho d\theta , \end{array}$$

where *f* (*c*, *r*) is the image function, and equation (13) is for digital images. The integral can be exchanged with the summation. Also, the image coordinates must be adjusted to [0,1] using mapping transformation.  Figure 4 depicts the mapping tranformation of the original image. Elements do not participate in the calculation of Z-moments.

The article "Multiresolution-Based Singular Value Decomposition Approach for Breast Cancer Image Classification" was retracted in 2024. Reasons: signs of a paper mill; suspected computer-generated content; unreliable results or conclusions; concerns about the data.

The discrete formal representation of Z-moments of an image is as follows:

(14) $$\begin{array}{c} Z_{n,m}=\frac{n+1}{\lambda \pi }\overset{N-1}{\underset{c=0}{\sum }}\overset{N-1}{\underset{r=0}{\sum }}f\left(c,r\right)V_{n,m}^{*}\left(c,r\right)=\frac{n+1}{\lambda \pi }\overset{N-1}{\underset{c=0}{\sum }}\overset{N-1}{\underset{r=0}{\sum }}f\left(c,r\right)R_{n,m}\left(\rho_{c,r}\right)e^{-jm\theta_{cr}}, \end{array}$$

where 0 ≤ *ρcr* ≤ 1 and *λπ* are normalization factors, in Z-moments. Transform distance *ρcr* and phase *θcr* at pixel (*c*, *r*) are given by the following formula [27]. Note that *c* and *r* represent the number of columns and rows.

(15) $$\begin{array}{c} \left\{\begin{array}{c} \rho_{cr}=\frac{\sqrt{{\left(2c-N+1\right)}^{2}+{\left(2r-N+1\right)}^{2}}}{N},\\ \theta_{cr}=\tan^{-1}\left(\frac{N-1-2r}{2c-N+1}\right). \end{array}\right. \end{array}$$

Using equations (14) and (15), we get only *c*, *r*, *m* and *n* in the final equation of the function. In fact, if the image ROI (region of interest) area has an odd number of rows and columns, it will have focal points as follows:

(16) $$\begin{array}{c} \left(c,r\right)=\left(\frac{N-1}{2},\frac{N-1}{2}\right). \end{array}$$

Combining equations (15) and (16), the following initial values can be obtained:

(17) $$\begin{array}{c} \left\{\begin{array}{c} \rho_{cr}=0,\\ \theta_{cr}=\tan^{-1}\left(\frac{0}{0}\right)=\text{Nan}. \end{array}\right. \end{array}$$

This paper chooses high-order Z-moments, although compared to low-order Z-moments, higher-order Z-moments not only have higher computational complexity degrees but also higher sensitivity to noise, so if there is no precise selection, system performance may degrade. However, due to the fact that high-order Z-moments describe shapes better than lower-order Z-moments and edge features, in order to more accurately analyze the contour of the image, this paper selects high-order Z-moments.

The article "Multiresolution-Based Singular Value Decomposition Approach for Breast Cancer Image Classification" was retracted in 2024. Reasons: signs of a paper mill; suspected computer-generated content; unreliable results or conclusions; concerns about the data.

By the values of *n* and *m* given in Table 1, it can be obtained from each low-frequency map, Z-moments consisting of 32 values are obtained from images or high-frequency images.

### 4.4. Classification of Support Vector Machines

There are many classification algorithms; this paper uses a support vector machine (SVM) classification method, because through experimental analysis, the classification effect of using SVM is the most. And through the feature extraction process of Z-moments, each original features are considered. The original mammogram has 32 × 15 = 480 features, but not all features are useful for image classification, so use the SVD method to reduce features and extract features that can represent more than 95% of the population. The top *K* values of the image information were obtained. This reduces the amount of data and shortens the classification training time, and the classification accuracy is improved. The idea of SVM is to map the input vector to a high-dimensional feature space, and then, the optimal classification surface is constructed in this high-dimensional space, which is originally linear and inseparable. The problem is transformed into a linearly separable one in high-dimensional space. At the same time, to avoid the “curse of dimensionality” from occurring, the kernel function *K* (*x*_*i*_, *x*_*j*_) = *ϕ*(*x*_*i*_)*ϕ*(*x*_*j*_) generation substitutes the inner product operation.

SVM cleverly solves high-dimensional and nonlinear problems and has good generalization, and there is a unique solution.  Algorithm 1 is the algorithm flow of SVM.

## 5. Experimental Setup and Result Analysis

### 5.1. Dataset

This article uses the 255 IRMA database of fatty breast tissue images, including 233 normal cases (no lesions), 72 benign cases, and 83 malignant cases [10]. The IRMA dataset documentation not only is detailed but also introduces the scanning methods for each mammography imaging and whether the imaging direction is the right breast or the left breast; the breast lesions are determined according to the standard classification of BIRADS: benign, malignant, and normal [24]. However, artifacts are often present in mammograms, such as by finger common grooves and grease caused by striations, which will make the image processing difficult. The IRMA database is selected through the use of specialized clinical knowledge; select a region of interest (ROI) to avoid these situations.  Figure 5 shows the 8 original breast images in IRMA with left and right sides and a comparison chart in the same direction. The IRMA medical image database also provides mammograms for calcifications, structural distortions, and asymmetries [29]. However, this paper only deals with mammograms that deal with fatty breast tissue picture. Additionally, using the IRMA database for classification applications, the dataset must also be balanced, so this experiment also synthesized 161 good sex cases and 150 malignant instances. The synthetic method is based on real graphs.

The article "Multiresolution-Based Singular Value Decomposition Approach for Breast Cancer Image Classification" was retracted in 2024. Reasons: signs of a paper mill; suspected computer-generated content; unreliable results or conclusions; concerns about the data.

Cancer develops when healthy breast cells change and expand uncontrollably, forming a mass or sheet of cells known as a tumor. A tumor may be cancerous or benign. A malignant tumor is one that can grow and spread to other areas of the body. A benign tumor is one that is able to develop but has not spread. This covers both noninvasive breast cancer (stage 0) and locally progressed and early-stage invasive breast cancer (stages I, II, and III) [21]. The breast cancer stage describes the size and spread of the tumor. Although breast cancer typically spreads to nearby lymph nodes, in which case it is still considered a local or regional disease, it can also move through the blood arteries and/or lymph nodes to the bones, lungs, liver, and brain. This is the most advanced stage of breast cancer, defined as stage IV or metastatic illness. However, lymph node involvement alone is often insufficient to diagnose breast cancer at stage IV [30].

### 5.2. Experimental Results and Analysis

To validate the classification method of NSCT-based mammography images, this paper mainly compares the experimental results of authors. Therefore, the experiment uses different classifiers or the same classification with different kernel functions of the processor, combining various processing processes to form a ratio that is more experimental.

Table 2 lists various experimental methods. Among them, the experimental formula and black method is the combination method proposed in this paper; there are 4 kinds in total, and the next will be based on these 4 types that are used to analyze experimental results.

#### 5.2.1. Analysis of Test Set Accuracy

Based on the 16 experimental schemes in Table 2, this paper first considers the accuracy of the test set classification results, which can also intuitively explain that this paper method outperforms other methods.

The article "Multiresolution-Based Singular Value Decomposition Approach for Breast Cancer Image Classification" was retracted in 2024. Reasons: signs of a paper mill; suspected computer-generated content; unreliable results or conclusions; concerns about the data.

As can be seen from Figure 6, for the kernel function of SVM, whether it is using linear, polynomial, RBF, or decision trees, the accuracy of the methodology is higher. For Sidney's 3 different discrete wavelet transforms, choosing the effect of Symlet8 waves is best among various classification methods. In addition, for this experiment, the kernel function of SVM has better performance when choosing linear and polynomial. Experimental results are good, and the experimental results of the linear kernel function are better.  Table 3 shows the accuracy of the test set.

#### 5.2.2. Temporal Analysis of the Training Set

While focusing on experimental accuracy, time efficiency is also an ignored metric. A good classification method needs to comprehensively consider accurate rate and time efficiency, balancing the two indicators to maximize the classification effect. It is more likely to be applied in practice if it is excellent.  Figure 7 and Table 4 give training time for various classification methods. It can be seen from Figure 7 that no matter which kind of classification method is adopted in this paper (class methods), the training time required for the training set is significantly lower than that of Sidney et al. who proposed 3 types of wavelet transforms. The reason is that unlike the method proposed by Sidney et al., the method in this paper performed first the singular value decomposition of the data, instead of directly using the resulting data as input to various classifiers, thereby reducing the dimension of the data and improving the efficiency of training time. Therefore, the method in this paper is to a certain extent practical.

In conclusion, 16 experimental methods of 4 types are implemented in this paper in the method, whether it is the experimental method proposed in this paper or literature. The proposed experimental method, the linear kernel function method of SVM, has achieved the best classification effect. And for the exploit proposed by literature, discrete wavelet transform decomposes images and also does a small comparative experiment of wave transform, and the experimental effect is expressed; Sidney et al. proposed the Symlet8-type discrete wavelet transform which has the best experimental results, but it is not as good as the NSCT method proposed in this paper. It is mainly due to the high-order Zernike moments which are used in the feature extraction stage, which are better than those of the authors. The low-order Zernike moments used by humans can extract more representative milk features of glandular X-ray images and be decomposed by SVD to make the features more representative, the amount of data is greatly reduced, and the time efficiency is also greatly improved.

The article "Multiresolution-Based Singular Value Decomposition Approach for Breast Cancer Image Classification" was retracted in 2024. Reasons: signs of a paper mill; suspected computer-generated content; unreliable results or conclusions; concerns about the data.

The proposed algorithm has been compared with the current state-of-the-art techniques. The methods include Biorthogonals3.8, Daubechies9, and Symlet9. The classification techniques used are SVM linear, SVM polynomial, SVM RFB, and decision tree. The accuracy of the proposed methodology is higher, i.e., 96.76%. It is also evident from the results obtained that the kernel function of SVM has better performance when choosing linear and polynomial.

## 6. Conclusion

This paper presents a classification method of mammography images based on NSCT. The method first decomposes the region of interest of the mammography image into multiresolution submaps through NSCT decomposition and then uses the Nick moment to extract the features in the subgraph, and in the data preprocessing stage, singular value decomposition is selected to reduce the features, so as to extract important features that can generalize globally. The method in this paper combines texture and shape features and uses an SVM-based classification algorithm to classify mammography images into normal, benign, and malignant and realizes the detection and classification of breast lesions. Taking into account the BIRADS criteria, this paper defines the categories of interest as normal (undamaged breast tissue), benign, and malignant lesions. Through the theoretical basis of mathematical morphology, it is proven that the mode spectrum is the ideal and unique shape representation of the binary image. And this paper also conducts feature extraction experiments using morphological spectroscopy and evaluates them. The experimental procedure combines 16 different algorithms of 4 types of classification methods.

More difficult mammography images such as dense, extremely dense, and fibroglandular breast tissue can be processed to a large extent based on the ideas of the method in this paper. With future improvements, it can also be applied to other forms of cancer diagnosis or other related biomedical image classification problems, such as brain magnetic resonance imaging, immunohistochemical images, and other complex image analysis problems where both morphology and texture are essential. The overall accuracy of the classification method in this paper is high, and the training time is relatively low, which is convenient for rapid promotion and helps doctors accurately diagnose the disease.

## Figures and Tables

**Figure 1:** Overall frame.

**Figure 2:** NSPFB decomposition process.

**Figure 3:** NSDFB decomposition process.

The article "Multiresolution-Based Singular Value Decomposition Approach for Breast Cancer Image Classification" was retracted in 2024. Reasons: signs of a paper mill; suspected computer-generated content; unreliable results or conclusions; concerns about the data.

**Figure 4:** Original image normalized map.

**Figure 5:** Original breast image.

**Figure 6:** Graphical analysis of accuracy of the test set.

**Figure 7:** Graphical analysis of training time.

**Algorithm 1:** SVM-based classification method.

**Table 1:** Higher-order Z-moment values of *n* and *m*.

*n*	*m*	Z-moment quantity
10	2,6,10	32
11	3,7,11	
12	0,6,8,10	
13	1,5,7,13	
14	2,6,8,16	
15	3,7,9,15	
16	0,2,4,14,16	
17	1,5,9,15,17	

**Table 2:** Experimental methods.

Method name	Classification	Feature extraction	Image decomposition
SVMI1	SVM linear	Higher-order Zernike moments, SVD	NSCT
SVMI2	SVM linear	Low-order Zernike moments	Biorthogonals3.8
SVMI3	SVM linear	Low-order Zernike moments	Daubechies9
SVMI4	SVM linear	Low-order Zernike moments	Symlet9
SVMp5	SVM polynomial	Higher-order Zernike moments, SVD	NSCT
SVMp6	SVM polynomial	Low-order Zernike moments	Biorthogonals3.8
SVMp7	SVM polynomial	Low-order Zernike moments	Daubechies9
SVMp8	SVM polynomial	Low-order Zernike moments	Symlet9
SVMR9	SVM RFB	Higher-order Zernike moments, SVD	NSCT
SVMR10	SVM RFB	Low-order Zernike moments	Biorthogonals3.8
SVMR11	SVM RFB	Low-order Zernike moments	Daubechies9
SVMR12	SVM RFB	Low-order Zernike moments	Symlet9
DT13	Decision tree	Higher-order Zernike moments, SVD	NSCT
DT14	Decision tree	Low-order Zernike moments	Biorthogonals3.8
DT15	Decision tree	Low-order Zernike moments	Daubechies9
DT16	Decision tree	Low-order Zernike moments	Symlet9

**Table 3:** Accuracy of the test set.

Test set precise rate (%)	SVM linear	SVM polynomial	SVM RFB	Decision tree
0	95	95	38	75
20	88	88	35	70
40	85	85	37	68
60	86	86	38	60
80	82	82	40	65

**Table 4:** Training time.

Train time (s)	SVM linear	SVM polynomial	SVM RFB	Decision tree
0	0.1	0.1	0.09	0.08
0.2	0.2	0.15	0.135	0.12
0.4	0.7	0.5	0.45	0.4
0.6	0.9	0.6	0.54	0.48
0.8	1	0.7	0.63	0.56
1.2	1.4	1	0.9	0.8
1.8	1.5	1.1	0.99	0.88
2	2	1.2	1.08	0.96

## Data Availability

The data shall be made available on request.
